The article "Recognition of Protein Network for Bioinformatics Knowledge Analysis Using Support Vector Machine" was retracted in 2024. Reasons: signs of a paper mill; suspected computer-generated content; unreliable results or conclusions; concerns about the data.

# Recognition of Protein Network for Bioinformatics Knowledge Analysis Using Support Vector Machine

**DOI:** 10.1155/2022/2273648

**Published:** 2022-04-23

**Authors:** Arshpreet Kaur, Abhijit Chitre, Kirti Wanjale, Pankaj Kumar, Shahajan Miah, Arnold C. Alguno

**Affiliations:** ^1^GNA University, Village Hargobindgarh, Phagwara, Punjab, India; ^2^Department of Electronics and Telecommunications, Vishwakarma Institute of Information Technology, Savitribai Phule Pune University, Pune, Maharashtra, India; ^3^Department of Computer Engineering, Vishwakarma Institute of Information Technology, Savitribai Phule Pune University, Pune, Maharashtra, India; ^4^Department of Computer Science & Engineering, Lloyd Institute of Engineering & Technology, Greater Noida, 201306 Uttar Pradesh, India; ^5^Department of EEE, Bangladesh University of Business and Technology (BUBT), Dhaka, Bangladesh; ^6^Department of Physics, Mindanao State University-Iligan Institute of Technology, Tibanga Highway, Iligan City 9200, Philippines

## Abstract

Protein is the material foundation of living things, and it directly takes part in and runs the process of living things itself. Predicting protein complexes helps us understand the structure and function of complexes, and it is an important foundation for studying how cells work. Genome-wide protein interaction (PPI) data is growing as high-throughput experiments become more common. The aim of this research is that it provides a dual-tree complex wavelet transform which is used to find out about the structure of proteins. It also identifies the secondary structure of protein network. Many computer-based methods for predicting protein complexes have also been developed in the field. Identifying the secondary structure of a protein is very important when you are studying protein characteristics and properties. This is how the protein sequence is added to the distance matrix. The scope of this research is that it can confidently predict certain protein complexes rapidly, which compensates for shortcomings in biological research. The three-dimensional coordinates of C atom are used to do this. According to the texture information in the distance matrix, the matrix is broken down into four levels by the double-tree complex wavelet transform because it has four levels. The subband energy and standard deviation in different directions are taken, and then, the two-dimensional feature vector is used to show the secondary structure features of the protein in a way that is easy to understand. Then, the KNN and SVM classifiers are used to classify the features that were found. Experiments show that a new feature called a dual-tree complex wavelet can improve the texture granularity and directionality of the traditional feature extraction method, which is called secondary structure.

## 1. Introduction

Protein is an important part of living things because it is made up of 20 types of natural amino acids. Proteins have different secondary structures because the order and number of these amino acids make them unique. Proposals for a classification of protein structures in the literature say that proteins are usually broken down into three main groups: A protein's secondary structure can be broken down into four groups: All-I, All-I, All-I, and All-I+I. The classification of secondary structure is important for more in-depth study of protein tertiary structure and how proteins work together. There has been a big rise in the size of protein databases over the last few years, but experimental annotation of protein structure classification has not kept up. So, there is a real need to make it easier to predict which structural proteins will be found and which ones will not.

Proteins are the building blocks of life. They are found in all living cells and play a role in almost all of life's activities. Because most proteins do not do their job alone, they work together with other proteins to form protein complexes [1]. As a result, predicting protein complexes helps us learn more about how cells and their processes work [2, 3]. The most important contribution of this research is that it contributes to show the extraction of secondary structure features of protein network. The dual-tree complex wavelet transform is employed for textural information in the distance matrix of proteins because it has strong direction selection and very little redundant data.

Some experimental techniques, like tandem affinity purification and mass spectrometry (TAP-MS) [4, 5] and yeast two-hybrid (Y2H) [6, 7], can directly detect protein complexes. However, the experimental results are not only different, but they also do not always agree. Because of the way nonsteady protein complexes move around, it can be hard to find less-addressed proteins again after multiple washes in tandem affinity purification and mass spectrometry experiments, because the less-addressed protein cannot be found again after many washes. The interactions between proteins are very complex and hard to detect with experiments. Some complexes can only be made in a specific environment, and if practical biological processes cannot recreate that environment, the complexes will not be found. Because it is hard to get the time, space, and other information about how proteins interact, this will also affect the accuracy of complex detection. Experiments in biology take a long time and cost a lot, which cannot meet the needs of research in the postgenome era.

With the rise of high-throughput experiments, more and more data about protein-protein interactions (PPI) is being collected every day. This makes it easier to predict protein complexes by using computational methods. Because there are many problems with biological experiment technology, computational methods are being used more and more in this field. They are good because they are fast and cheap. They can quickly predict some protein complexes with a high level of confidence, which makes up for the flaws in biological experiments [8, 9]. There are various effects of excess use of protein in human body. It may place an oxidative acidosis mostly on joints, kidneys, and heart. Furthermore, elevated foods may be implicated in the development of cardiovascular disease or possibly cancer owing to excessive blood pressure and cholesterol levels consumption. There are many ways to make a network of proteins that interact with each other. For example, you can use a lot of data about how proteins interact with each other. Among them, the nodes in the network are proteins, and the connections between them show how the proteins interact with each other. Then, complex network theory and machine learning can be used to figure out what protein complexes will look like on PINs.

There are usually two steps to figuring out how proteins will look in the future. In the first place, proteins of different lengths can be represented by feature vectors of the same length through feature extraction. Then, the feature vectors are put into a specific algorithm for making predictions. Mathematical, statistical, and spectral analysis methods have been used to look at protein sequence features. These methods include amino acid composition characteristics [2, 3], pseudoamino acid composition [3, 4], dipeptide and polypeptide composition [4, 5], multiple evolutionary matrices [6, 7], gene sequence information [10, 11], and fusion of different features, for example. Amino acids are the building blocks of proteins. These acids have no color. Proteins have distinct secondary structures according to the order and amount of amino acids in each one. According to statistics and machine learning, a lot of different ways to predict what will happen have been developed. The KNN method is a basic automated computational model that is being used to handle classification and regression issues. It is simple to use and comprehend. It is easy to put into exercise and comprehend. These include the nearest neighbor method (KNN), hidden Markov model (HMM), Bayesian network, artificial neural network, and support vector machine (SVM) [8–12].

After converting the protein sequence into a distance matrix, it can be seen that it looks like a texture picture. Grey-level cooccurrence matrix and grey-level histogram statistics are used to figure out what it looks like. In this research, the authors have used computational methods for the prediction of protein complexes. The future scope of this proposed method is that it can confidently predict certain protein complexes rapidly, which compensates for shortcomings in biological research. However, the result of the input classifier's classification is not the same. Using the wavelet transform, this paper comes up with a way to get the features out of the distance matrix. The dual-tree complex wavelet transform was created to solve some problems with the traditional dimensional discrete real wavelet transform in image processing [13, 14]. It has been used to get good results in image processing [13, 14]. This is called the dual-tree complex wavelet transform. It uses two pairs of filter banks to do the L-level decomposition of the image.

Furthermore, it uses the six directional subbands that were found at each scale to figure out their energies and standard deviations and build feature vectors based on that. The double-tree complex wavelet transform is used in this paper to finish extracting the features from the transformed protein distance matrix. The following sections show that this method is very good at classifying proteins with secondary structures.

The present article has been planned into six sections. The introduction is described in Section 1.  Section 2 puts light on protein structure and their predictions.  Section 3 described computation-based methods for protein complex prediction. Prediction algorithm based on weighted network is described in Section 3.3. The materials and methods are described in Section 4. Comparative result analysis is described in Section 5; finally, Section 6 portrays the conclusion and possible future works based on the proposed framework.

## 2. Protein Structure and Their Predictions

A protein complex is a collection of proteins that gather together to complete a specific biological function or biological process by interacting with each other at a particular time and space. Therefore, protein complexes play a crucial role in the normal functioning of organisms. Common protein complexes include RNA polymerase for RNA synthesis during transcription and proteasome for molecular degradation.  Figure 1 shows the new coronavirus RNA-dependent RNA polymerase [13] (PDB ID: 6M71), the core component of the new coronavirus transcription and replication and is considered an essential antiviral drug target. Sivir is an antiviral drug based on this target. Different colors in the figure represent other peptide chains; green, orange, purple, and blue represent the A chain, B chain, C chain, and D chain in the complex, respectively. The interaction between different chains constitutes a protein complex.

Biological methods for detecting protein complexes mainly include tandem affinity purification, mass spectrometry technology, and yeast two-hybrid technology. Below, these two biological methods are briefly introduced.

Tandem affinity purification and mass spectrometry are essential tools in current proteomics research. The primary step is to embed a protein tag and introduce the target protein. The proteins that interact with the target protein under physiological conditions can be eluted together and then identified by mass spectrometry technology. The natural conditions under physiological conditions can be quickly obtained protein complexes [4, 5].

Yeast two-hybrid technology detects protein complexes. First, the known coding protein DNA sequence is ligated to an expression vector with transcriptional regulator DNA; then, the introduced yeast cells are combined with the promoter region upstream of the reporter gene. Next, as a “bait” protein, the DNA known to encode the transcription activation domain is ligated with different fragments in the cDNA library to be screened to obtain a “prey” vector; finally, the reporter gene expression is activated, and a protein complex is obtained [6, 7].

It is possible to look at protein complexes directly with techniques like tandem affinity purification, mass spectrometry, and yeast two-hybrid, but there are a lot of false positives and false negatives in the results. Some protein complexes are also hard to find because of the limitations of practical technology. In the postgenome era, there are problems that cannot be solved because they take a long time and cost a lot of money. With the rise of high-throughput experiments, the amount of information about how many different kinds of proteins interact with each other across the whole genome has grown. This has made it easier for computer programs to predict protein complexes.

For example, computer-based methods for predicting how proteins work together can make up for the inaccuracies in biological experiments. There are a lot of high-confidence protein complexes that can be found on large biological networks very quickly. In the current computer programs, the relationship between proteins is usually shown as a network that does not go anywhere. This is called G = (V, E). All three of these things are called “G,” “V,” and “E.” They all refer to the protein interaction network, “V,” and “E.” Figure 2 shows how the yeast proteins interact with each other. The protein-protein interaction (PPI) makes computer approaches for predicting protein structures easier. Although biological experimental technique has so many flaws, analytical techniques are increasingly being applied in this sector. They are beneficial since they are quick and inexpensive. The calculation-based method predicts protein complexes by looking at the topology structure of the network and the biological properties of the nodes as features. The clustering method is used to find the dense subgraph on the PPI network, and the dense subgraph is used as the final dense subgraph. The results show that the computationally based method can be used to look at PPI networks, predict protein complexes, and more.

## 3. Computation-Based Methods for Protein Complex Prediction

At the moment, both domestic and foreign scientists have come up with a number of computer-based algorithms for predicting the structure of protein complexes. This paper breaks down these methods into the following seven groups: based on dense subgraphs, prediction algorithms based on the core-subsidiary structure, and algorithms that use dynamic networks to predict what will happen, learning algorithms that use supervised learning, algorithms that move from function to interaction, algorithms that use data from multiple sources, and other methods can be used to make predictions about how people will act together.

### 3.1. Prediction Algorithms Based on Local Dense Subgraphs

There are seven types of algorithms for making predictions. The algorithms based on local dense subgraphs are the oldest and most common of these seven types. Because most proteins need to work together to form complexes to do their jobs in the body, the proteomes in the complexes are nodes in the interaction network, or dense subgraphs. Protein interaction networks have been shown to be modular by a lot of different studies [4, 5].

Network topology shows that modules in a PPI network are made up of proteins that are close together. From a biological point of view, modules in a PPI network are groups of proteins that work together to perform a specific biological task. When you look at the modular structure (i.e., dense subgraphs or subnetworks) in the PPI network, you can figure out what kinds of protein complexes are likely. If the edges in the PPI network are weighted, methods based on dense subgraphs can be broken down into two groups: algorithms based on unweighted networks and algorithms based on additive networks.

### 3.2. Prediction Algorithm Based on Unweighted Network

In 2003, Bader and Hogue came up with the MCODE [15] method, which was one of the first computational methods for predicting protein complexes. It does this in three steps. To figure out a node's local neighbor density, you first need to figure out its k-core value and the density of its local subgraph. Then, choose the node with the highest density value as the seed node. Then, go through its neighbors and expand, and add the nodes that meet the corresponding threshold to the current subgraph in turn, until the subgraph no longer grows and the first protein is found complex. Afterward, nodes that have not been processed are used as new seed nodes, and the same thing happens again. Finally, to improve the accuracy of the predictions, MCODE does some postprocessing on the above-predicted initial complexes. There are two ways to get rid of complexes with less than two nodes: for each node v in the candidate complex, if the density of the subgraph formed by its direct neighbors (including node v) is higher than a given parameter, then all the nodes of v's direct neighbors are added to the current complex in turn and the final protein complexes are made, as shown in the figure.

Network-based clustering algorithms have been used to look for dense subgraphs in protein interaction networks that are likely to be protein complexes [12–17]. For example, the MCL algorithm takes the dense subgraphs from the graphs to predict protein complexes. The random walk keeps doing the two operations of “expanding” and “expanding” on the adjacency matrix that was made by the PPI network. This makes the dense area in the PPI network more viscous and the sparse area sparser so that the closely connected node group is used as the compound output. Because the algorithm does matrix operations right away, it is a fast and scalable clustering algorithm [17].

### 3.3. Prediction Algorithm Based on Weighted Network

When we look at unweighted protein interaction networks, you only look at whether there is a relationship between two proteins. False positives and false negatives are found in the protein interaction data because of the incompleteness of current biological experiments. Liu et al. devised a method for grouping items associated with the entire graph. The weight of the relevant edge is determined first by the number of known neighbors the node has. This value is then modified repeatedly. The PPI network's whole graph is then identified, and the weight of each edge is determined. This is completed next. Finally, assemble them into a complex based on their scores. The confidence in the unweighted network that was built by this is also low. Because of this, some studies have made the PPI network more reliable by putting more weight on the edges of the PPI network topology, gene expression data, protein function, and other information, and on this basis, they came up with a weighted network-based complex prediction algorithm.

Weighted networks were made in the early days by figuring out how many proteins that interact with each other have neighbors who know each other [3]. Literature came up with the DPClus algorithm, which assigns edges between node pairs based on the number of people who know each other. The weight of a node is the sum of the effects of the edges that are next to it. Use the node with the most significant weight as the seed and the clustering attribute to add nodes that are more connected to their neighbors into the cluster, which is called a cluster. In addition, literature [18] made changes based on DPClus and came up with a new way to predict protein complexes. Liu et al. came up with a way to group things together based on the full complete graph. The weight of the corresponding edge is first measured by how many familiar neighbors the node has. This value is then changed over and over again. Then, the full graph in the PPI network is found, and the weight of each edge is calculated. This is done next. Finally, put them together based on their scores to make a complex. In the beginning, weighted networks were created by calculating how many proteins that interacted with each other had neighbors that know each other. The literature [13] algorithm makes a directed weighted graph based on the number of proteins that are close to each other. First, the protein with the highest degree is chosen to be the core of the first layer. Then, the nodes with weights above a certain threshold are connected to the core of the first layer. This is then linked to making a second layer of the core and, finally, expanding to make the last protein complex. Literature [12] also used the number of proteins that are close to each other as an edge weight. They came up with the WN-PC method to predict protein complexes. Literature [14] uses the spoke model to make clusters based on the types of nodes and how important they are. These clusters are then combined based on cohesion to make the final protein complexes. Literature [16] sets a threshold based on the weighted density of the complex and the size of the cluster. It then uses a strategy similar to DPClus to make complexes, which can quickly cluster large biological networks.

## 4. Materials and Methods

### 4.1. Datasets

Two datasets are used in this paper, from the literature [16] and literature [15], respectively. The PDB database has the three-dimensional coordinates of C*α* atoms of protein sequences in both datasets. In the process of downloading the data, it was found that some protein data in the literature did not exist in the PDB database, so this paper selected the complete protein sequence of the three-dimensional data of the C*α* atom and finally obtained the first dataset containing a total of 197 proteins, of which 48 All-*α* class, 60 All-*β*, 45 *α β* class, and 44 *α*+*β* class, from now on referred to as dataset A; the second dataset contains a total of 1 656 proteins, of which 440 All-*α* class, 437 All-beta classes, 342 alpha-beta classes, and 437 alpha+beta classes, after this referred to as dataset B. The secondary structure data of each protein contained in the two datasets are shown in Table 1.

### 4.2. Texture Information in the Distance Matrix

The key to establishing the prediction method is to extract the protein sequence features and use the protein backbone to describe its secondary structure, that is, use the three-dimensional coordinates of the C*α* atoms to calculate the distance between all C*α* atoms on each protein chain to form a matrix, so that the matrix contains sufficient 3D structural information of the protein structure in addition to the chirality [17]. Therefore, the features of the protein distance matrix can be extracted to compare the 3D structure of the protein.

Let the protein sequence psi of length *L* be

(1) $$\begin{array}{c} {\text{ps}}_{\text{i}}=r_{1},r_{2},\cdots \cdots r_{n}, \end{array}$$

where *r*_1_, *r*_2_, ⋯*r*_*n*_ represents the protein sequence Psi amino acid residues. So then, its skeleton can be defined as

(2) $$\begin{array}{c} \beta_{i}=\left\{c_{\alpha 1}^{i},c_{\alpha 2}^{i},c_{\alpha 3}^{i},\cdots \cdots .c_{\alpha l}^{i}\right\}, \end{array}$$

where *c*_*αl*_^*i*^ is the three-dimensional coordinate vector of the C*α* atom of the L^th^ amino acid residue, and then the protein sequence Pi is converted into a distance matrix DM = {dmi(m, n) = dist(*c*_*αn*_^*i*^, *c*_*αm*_^*i*^)1 ≤ m, n ≤ L}, where dist is the Euclidean distance.

In this paper, the distance matrix of proteins is regarded as a texture image; that is, each element in the matrix corresponds to an image pixel, and the value of each element is mapped to the grey value of the corresponding pixel. It can be seen from Figure 3 that the grayscale images of the four different protein structure types are completely different, and they have very different texture features, so the information in the distance matrix can be extracted by image processing so that the protein sequences are converted into feature vectors of a certain dimension.

The texture is important information and feature of an image, and it is an effective method to use the texture feature of an image to classify. The methods of extracting image texture features include grayscale histogram, grayscale cooccurrence matrix, and wavelet transform-based methods. Still, the grayscale histogram of the image only counts the first-order information of the picture, and the grayscale cooccurrence matrix only describes the coarse granularity. Because of the texture characteristics, two-dimensional wavelet transform has the defects of translation change and limited direction selectivity. The dual-tree complex wavelet transform proposed by Kingsbury [19] has approximate translation invariance, good direction selectivity, and little data redundancy. Therefore, it can extract image features from different directions and enrich texture information. The texture of an image is crucial information and a feature, and using the texture feature of an image to classify is an effective way. The feature extraction method plays an important role for the extraction of protein features. The approaches for feature extraction are useful in a variety of image enhancement, such as feature segmentation. The disadvantage of image retrieval has been that the new features created are incomprehensible to individuals.

### 4.3. Dual-Tree Complex Wavelet Features

The two-dimensional dual-tree complex wavelet is defined as

(3) $$\begin{array}{c} \varphi^{\text{c}}\left(\text{p},\text{q}\right)=\left[\vartheta_{\text{i}}\left(\text{p}\right)+{\text{k}\vartheta }_{\text{j}}\left(\text{p}\right)\right]\left[\vartheta_{\text{i}}\left(\text{q}\right)+{\text{k}\vartheta }_{\text{j}}\left(\text{q}\right)\right], \end{array}$$

where *i* is an imaginary number, *i*^2^ = −1, and *ϑ*_*i*_ and *ϑ*_*j*_ are orthogonal or biorthogonal real wavelets, respectively, and form a pair of Hibert transforms. Dual-tree complex wavelet transform can be implemented by discrete wavelet transform DWT, one DWT produces the real part and the other DWT produces the imaginary part. Its decomposition process is shown in Figure 4.

As can be seen from Figure 4, the dual-tree complex wavelet transform essentially uses two sets of low-pass filters i0(n), j0(n) and high-pass filters i1(n), j1(n) to transform the input two-dimensional. The signal is alternately transformed between rows and columns, and 2 low-frequency subbands and 6 high-frequency subbands in different directions (-75°, -45°, -15°, 15°, 45°, and 75°) are decomposed. In this way, after the image is decomposed, its texture features can be analyzed from more directions. The higher the level of wavelet decomposition, the more detailed features in the multiscale image can be obtained, but if the decomposition level is too high, not only the boundary effect of the feature image will be more obvious, affecting the classification accuracy, but also the calculation of wavelet transform will be increased. Therefore, in this paper, the distance matrix is decomposed by a 4-level dual-tree complex wavelet, and there are 6 directional subbands *W*_ln_(*i*, *j*) at each scale, where *l* = 1,2,3,4, and *n* = 1, 2,3,4,5,6. Calculate the energy El, *n*, and the standard deviation *σ* according to equations (4) and (5) for these 6 subbands.

(4) $$\begin{array}{c} e_{\ln}=\frac{1}{\text{mn}}\overset{m}{\underset{i=1}{\sum }}\overset{n}{\underset{i=1}{\sum }}w_{\ln}\left(i,j\right), \end{array}$$

(5) $$\begin{array}{c} \sigma_{\text{in}}={\left[\frac{1}{\text{mn}}\overset{m}{\underset{i=1}{\sum }}\overset{n}{\underset{i=1}{\sum }}\;{\left(w_{\ln}\left(i,j\right)-\mu_{\text{lm}}\right)}^{2}\right]}^{1/2}, \end{array}$$

where m × n is the size of the subband image *w*_ln_(*i*, *j*) and *μ*l, n is the mean of *w*_ln_(*i*, *j*). Using a combination of standard deviation and energy features, the following 48-dimensional feature vector is obtained:

(6) $$\begin{array}{c} f={\text{e}}_{1,1,}\sigma_{1,1}\cdots \cdots ..{\text{e}}_{1,6,}\sigma_{1,6}\cdots \cdots \cdots \cdots \cdots {\text{e}}_{4,1,}\sigma_{4,1}\cdots \cdots .{\text{e}}_{4,6,}\sigma_{4,6}. \end{array}$$

After the protein sequence is transformed through the above steps, a 48-dimensional feature vector *F* can be obtained for protein sequences of different lengths.

### 4.4. Classification Prediction

Extract the features of the proteins in the two datasets according to the above method, and input them into the KNN classifier, where *K* is 5. Tenfold cross-validation is adopted for each experiment, and the average value of the results of the five experiments is calculated as the final result. After calculating the two feature vectors, the normalized Euclidean distance metric method in [20] is used.

To test the prediction performance of the method, this paper adopts five indicators: sensitivity, specificity, accuracy, Mathew's correlation coefficient, and overall accuracies.

## 5. Comparative Result Analysis

To test the prediction performance of the method, this paper adopts five indicators: sensitivity, specificity, accuracy, Mathew's correlation coefficient, and overall accuracies.

According to those mentioned above dual-tree complex wavelet feature extraction and KNN classification method, the prediction results on datasets A and B are shown in Tables 2 and 3. It can be seen from Tables 2 and 3 that when using the dual-tree complex wavelet transform to extract the texture features of the distance matrix, the performance on both datasets is excellent, and most of the results of the four indicators range from 94% to 100%. On the two structural categories of All-*α* and All-*β* in dataset A, the specificity reaches 100%. This is because the dual-tree complex wavelet transform uses two trees to transform the image, enhancing texture information expression [21]. For the convenience of comparison, this paper also extracts other features of the distance matrix according to the following methods.

1. Extract the statistical features of the grey histogram [22]; that is, calculate the mean, variance, contrast, third-order central moment, fourth-order central moment, uniformity, and entropy of the image and obtain a 7-dimensional feature vector
2. Extract the grey-level cooccurrence matrix features; that is, calculate the grey-level cooccurrence matrix in the three directions of 0°, 45°, and 135° according to the distance matrix and then calculate the contrast, correlation, and energy of the grey-level cooccurrence matrix in each direction and uniformity of these four features, and finally get a 12-dimensional feature vector
3. Extract the wavelet energy feature; that is, use the sym4 wavelet packet to decompose the distance matrix in four levels and calculate the energy percentage Ea of the corresponding approximate coefficient and the corresponding horizontal detail coefficient Eh, vertical coefficient Ev, and diagonal detail coefficient energy percentage Ed; these results in a 13-dimensional feature vector. The above feature vectors are input into the KNN classifier, respectively, for classification, and the value of *K* in KNN is all 5. Tables 4 and 5 list the KNN classification results of the above four features extracted from datasets A and B, respectively

It can be seen from Tables 4 and 5 that the double-tree complex wavelet features of the distance matrix are extracted, and the overall classification accuracy rates on dataset A and dataset B are 89.33% and 99.87%, respectively, which are better than the grey-level histogram statistical features and grey-level cooccurrence [22]. The matrix features are much higher, and for each secondary structure classification, the accuracy is improved to varying degrees. In some structural categories, the dual-tree complex wavelet feature is slightly lower than the wavelet energy feature, but in general, the method in this paper is more reliable.

To prove that the effect of the feature extraction method in this paper does not depend on the classification algorithm, SVM classifier classification is also used in the experiment. With the help of an easy-to-use and fast and effective SVM software package LIBSVM developed and designed by Professor Lin Zhiren of the National Taiwan University, the SVM in main parameters (optimal penalty parameter c and kernel function parameter g) are obtained by grid search method, RBF is selected as the kernel function, ten-fold cross-validation is adopted in each experiment, and the average of five experimental results is calculated as the final result.

As can be seen from Table 4, using the SVM classifier classification, compared with the previous three feature representation methods, the dual-tree complex wavelet features are 7.15, 5.72, and 4.84 percentage points higher on dataset A, respectively, and the results on dataset B are 3.51, 1.69, and 0.53 percentage points higher, respectively. To more intuitively reflect the method's effectiveness in this paper, the overall accuracy of extracting features using different techniques on dataset A and dataset B is shown in Figures 5 and 6.

As can be seen from Figures 7 and 8, the accuracy of the extracted grayscale histogram statistical features and grayscale cooccurrence matrix features is generally lower than that of the extracted wavelet transform elements because the grayscale histogram is only removed from the first-order statistical information of the image which is difficult to reflect the spatial position of the image pixels and other related information. The grey-level cooccurrence matrix only describes the characteristics of the texture from a relatively coarse granularity. Therefore, it lacks the overall spatial distribution characteristics of the image texture. At the same time, the wavelet transform can decompose the image into multiple frequency bands and has directionality, fully mining the surface and details of the image information. The accuracy rate of using dual-tree complex wavelet transform is slightly higher than that of wavelet energy features, and this is because wavelet transform has two main disadvantages when processing images, namely, translation variability and limited orientation selectivity. In contrast, dual-tree complex wavelet transforms to solve these two problems; it can extract image information from different directions and enrich the features of the image.

## 6. Conclusion

In this paper, a dual-tree complex wavelet transform is used to find out about the structure of proteins. For the texture information in the distance matrix of proteins, the dual-tree complex wavelet transform is used because it has good direction selectivity and very little data redundancy. This study introduces a new feature known as a dual-tree complex wavelet, which improves the texture granularity and directionality of the standard feature extraction approach known as secondary structure. The dual-tree complex wavelet transform uses two trees to transform the image, enhancing texture information expression. It is important to avoid the problem that the grey cooccurrence matrix of a traditional extracted image does not show how the overall spatial distribution of the texture of the image looks, so KNN and SVM are used to classify the extracted feature vectors. Classification has been checked, and the prediction results look good. They reached 98.50 percent and 99.29 percent, respectively, when they used the SVM to classify the two datasets. There are a lot of ways to look for features in protein sequences, like the classic pseudoamino acid component method. When we look into the future, we can try to improve the traditional process, combine it with this method, and use it with protein data that has texture features.

## Figures and Tables

**Figure 1:** RNA polymerase.

**Figure 2:** Protein-protein interaction network.

**Figure 3:** Texture map of different protein secondary structures.

**Figure 4:** Decomposition of two-dimensional DT-CWT.

**Figure 5:** Performance prediction of proposed work over dataset A.

**Figure 6:** Performance prediction of proposed work over dataset B.

**Figure 7:** Comparative performance prediction over dataset A.

**Figure 8:** Comparative performance prediction over dataset B.

**Table 1:** Dataset.

Dataset	*α*	*β*	*α*/*β*	*α*+*β*	Total
A	48	60	45	44	197
B	440	437	342	437	1656

**Table 2:** Performance prediction of proposed work over dataset A.

Parameter	Proposed structure			
	*α*	*β*	*α*/*β*	*α+β*
Sensitivity	92.56	94.26	90.56	92.23
Specificity	95.56	96.28	93.45	94.12
Accuracy	96.45	98.56	94.62	95.68
MCC	94.24	96.45	92.12	93.58

**Table 3:** Performance prediction of proposed work over dataset B.

Parameter	Proposed structure			
	*α*	*β*	*α*/*β*	*α*+*β*
Sensitivity	95.45	93.41	89.45	93.41
Specificity	96.45	95.26	89.25	95.23
Accuracy	98.12	98.45	92.85	96.48
MCC	97.12	95.12	91.57	95.12

**Table 4:** Comparative performance prediction over dataset A.

Extract features	Proposed structure				
	*α*	*β*	*α*/*β*	*α*+*β*	OA
Grayscale histogram	78.56	79.23	75.23	85.68	86.78
Grey-level cooccurrence matrix	76.23	76.48	74.24	79.48	82.56
Wavelet energy	79.23	80.45	75.28	82.45	84.89
Double-tree complex wavelet	80.12	82.23	79.46	85.56	89.46

**Table 5:** Comparative performance prediction over dataset B.

Extract features	*α*	*β*	*α*/*β*	*α*+*β*	OA
Grayscale histogram	79.56	81.28	76.25	87.26	89.52
Grey-level cooccurrence matrix	77.42	77.98	75.68	89.26	92.12
Wavelet energy	80.56	82.4	78.26	84.56	88.45
Double-tree complex wavelet	81.89	83.47	80.45	89.26	90.12

## Data Availability

The data shall be made available on request.
